The article "Paederia foetida Linn. leaf extract: an antihyperlipidemic, antihyperglycaemic and antioxidant activity" was retracted in 2025. Reasons: duplicated images; overlap with earlier publications; concerns about the images.

# *Paederia foetida* Linn. leaf extract: an antihyperlipidemic, antihyperglycaemic and antioxidant activity

**DOI:** 10.1186/1472-6882-14-76

**Published:** 2014-02-25

**Authors:** Vikas Kumar, Firoz Anwar, Danish Ahmed, Amita Verma, Aftab Ahmed, Zoheir A Damanhouri, Vatsala Mishra, Pramod W Ramteke, Prakash Chandra Bhatt, Mohd Mujeeb

**Affiliations:** 1 Department of Pharmaceutical Sciences, Faculty of Health Sciences, Sam Higginbottom Institute of Agriculture, Technology & Sciences (SHIATS)-Deemed University, Allahabad, Uttar Pradesh 211007, India; 2 Sidharatha Institute of Pharmacy, Dehradun, Uttrakhand, India; 3 Health Information Technology Department, Jeddah Community College, King Abdulaziz University, Jeddah 21589, Kingdom of Saudi Arabia; 4 Department of Pharmacology, Faculty of Medicine, King Abdulaziz University, Jeddah, Saudi Arabia; 5 Department of Pathology, MLN Medical College Allahabad, Allahabad, Uttar Pradesh, India; 6 Department of Biological Sciences, Sam Higginbottom Institute of Agriculture, Technology & Sciences (SHIATS)-Deemed University, Allahabad, Uttar Pradesh, India; 7 Department of Phytochemisty & Pharmacognosym, Faculty of Pharmacy, Jamia Hamdard, New Delhi 110062, India

**Keywords:** *Paederia foetida*, Antihyperlipedemic, Hexokinase, Antioxidative

## Abstract

**Background:**

The primary objective of the present investigation is to evaluate the antidiabetic, antihyperlidemic and antioxidant activity of the methanolic extract of the *Paederia foetida* Linn. (*PF*) leaf extract in the streptozotocin induced diabetic rats.

**Methods:**

Single intraperitoneal injection (IP) of streptozotocin (60 mg/kg body weight) was used for induction of diabetes is swiss albino (wistar strain) rats. The induction of diabetes was confirmed after 3 days as noticing the increase in blood sugar level of tested rats. *PF* at a once a daily dose of 100 mg/kg, 250 mg/kg, 500 mg/kg, p.o. along with glibenclamide 10 mg/kg, p.o. was also given for 28 days. On the 28^th^ day rats from all the groups fasted overnight fasted and the blood was collected from the puncturing the retro orbit of the eye under mild anesthetic condition. There collected blood sample was used to determine the antihyperlipidemic, hypoglycemic and antioxidant parameters.

**Results:**

The oral acute toxicity studies did not show any toxic effect till the dose at 2000 mg/kg. While oral glucose tolerance test showed better glucose tolerance in tested rats. The statistical data indicated that the different dose of the *PF* significantly increased the body weight, hexokinase, plasma insulin, high density lipoprotein cholesterol, superoxide dismutase, catalase and glutathione peroxides. It also decreases the level of fasting blood glucose, total cholesterol, triglycerides, low density lipoprotein cholesterol, very low density lipoprotein cholesterol, malonaldehyde, glucose-6-phosphate, fructose-1-6-biphosphate and glycated hemoglobin in STZ induced diabetic rats. The histopathology of STZ induce diabetic rats, as expected the test dose of *PF* extract considerably modulates the pathological condition of various vital organ viz. heart, kidney, liver, pancreas as shown in the histopathology examinations.

The article "Paederia foetida Linn. leaf extract: an antihyperlipidemic, antihyperglycaemic and antioxidant activity" was retracted in 2025. Reasons: duplicated images; overlap with earlier publications; concerns about the images.

**Conclusions:**

Our investigation has clearly indicated that the leaf extract of *Paederia foetida* Linn. showed remarkable antihyperglycemic activity due to its possible systematic effect involving in the pancreatic and extra pancreatic mechanism. Forever, the antihyperlipidemic activity was exerted possible by lowering the higher level of lipid profile and decreasing the intercalated disc space in the heart. The antioxidant activity of extract was due to inhibition of lipid peroxidation and increasing the SOD, GPx and CAT. It was corroborate that the extract shown the *Paederia foetida* Linn leaves potential to be act as antidiabetic, antihyperlipidemic and antioxidant properties.

## Background

Diabetes mellitus (DM) is a condition in which the amount of glucose increases in the blood, because organs viz. adipose tissues and liver does not properly utilize the glucose. DM occurs due to hereditary and environmental causes, resulting in abnormally high blood sugar level [1,2]. The role of the insulin in the body it release after a meal from the pancreas and stimulate the fat cells and muscle to remove the glucose from the blood and stimulate the liver to metabolize glucose, causing the blood sugar level to decrease to normal level. According to the WHO (World Health Organization) an estimated 300 million during World, 57.2 million adults in India affected in the year 2025 [3,4]. DM is the most common manifestation of metabolic disorder occurs in human due to the high consumption of carbohydrates and lipids [5]. Hyperglycaemia an associate with hyperlipidemia in the late phase of life is also prone to diabetes [6]. It is the complex metabolic endocrine disorder which resulting from disequilibrium of dynamic expression, causing the macro (heart attack, stroke and peripheral vascular disease) and micro (retinopathy, neuropathy and nephropathy) vascular complications [7,8]. Further, increase in the blood glucose level in diabetic patient causes alteration in utilization of glucose in the vital organs viz. adipose tissues and liver of the body. Increased in blood glucose level continuously generating reactive oxygen species (ROS) and superoxide anions, which further aggravate the diabetic complication by damaging the protein, deoxyribosenucleic acid and carbohydrate, which leading to increasing the oxidative stress [9-12]. The concentration of free radical production could be favorably reduced through appropriate dietary intake and drug therapy and thus less chance of diabetes and diabetic associated CVS disorder. Since there is no current treatment available for hypoglycemic, hypolipidemic and antioxidant drug together therefore, researchers are continuously working on discovery of effective drug to exert the action on hyperglycemia, hyperlipidemia and antioxidant effect with minimal or no signs of side or toxic effects.

The article "Paederia foetida Linn. leaf extract: an antihyperlipidemic, antihyperglycaemic and antioxidant activity" was retracted in 2025. Reasons: duplicated images; overlap with earlier publications; concerns about the images.

Medicinal plants play as important role in the discovery of new counteractive agents and received much more attention as a source of biologically active substance including antioxidant, antihyperglycemic and antihyperlipidemic agents [13]. Since few decades, plants were used to treat diabetes and its complications. 400 plants and there 700 recipes in the formulation were used for the treatment of diabetes [14]. Consequently, modern medical science explores this fruitful field and thus discovered a first clinically used drug of its own kind from to treat diabetes i.e. metformin (*Galega officinalis*). By above investigation and the role of plant in generation of antidiabetic agents [15]. Present investigation carried out to evaluate the antidiabetic, antihyperlipidemic and antioxidant stress activity of *Paederia foetida* Linn.

*Paederia foetida* Linn. Belonging to family Rubiaceae, commonly known as *Ghandhali* in across the India and usually found upto an altitude 1800 m in Himalaya region. in folklore system of medicine it was indicated for the treatment of gout, diarrhea, piles, dysentery, calculi, stomachic, emetic, ulcers and different type of inflammations [16-19]. It has also been reported for antinocietive [20], antiviral [21], antidiarrhoeal [22], anti tussive [23], anti-inflammatory [24] and anti cancer activity [25]. It was reported that majority of chemical constituents were found in leaves of *Paederia foetida* Linn., these chemical constituents comprise of iridoid glycoside, sitosterol, alkaloids, carbohydrates, β-sitosterol, ascorbic acid, flavonoids, amino acids, stigmosterol, D/L galacturonic acid and volatile oil *Paederia foetida* Linn. [26-28]. The aim of the present study was to evaluate the antidiabetic, antihyperlipidemic and antioxidant activity of the methanolic extract of the *Paederia foetida* Linn. (*PF*) leaf extract in the STZ induced diabetic rats.

## Methods

### Plant materials

Fresh leaves of *Paederia foetida* Linn. was collected from Herbal garden, Department of Life Sciences, Dibrugarh University, Dibrugarh, Assam, India and authenticated by the Botanical Survey of India, Shillong, India. A voucher specimen (Ref. No.DU/PSc/HRB-2/08) was deposited for future reference.

The article "Paederia foetida Linn. leaf extract: an antihyperlipidemic, antihyperglycaemic and antioxidant activity" was retracted in 2025. Reasons: duplicated images; overlap with earlier publications; concerns about the images.

### Preparation of crude extracts

The collected leaves of *PF* were gently washed with tap water to remove the extraporeneous matter. After rinsing, the leaves were dried in shade at room temperature. The leaves were grounded and approximately 2 kg leaves were extracted with methanol in a Soxhlet apparatus for 5 days. The filtrate obtained after filtration of above mention extract was concentrated under reduced pressure at 4°C using rotatory evaporator until the extra solvent completely disappear resulting the crude semisolid residue (percentage yield, 30%). The resulting product was then stored at 4°C until further use. To carry out animal studies of this product, it was dissolved in 2% solution of CMC (Carboxyl methyl cellulose) in distilled water [28-30].

### Extract standardization by HPTLC technique

#### Preparation of standard and sample solution

A stock solution of quercetin and ascorbic acid was prepared by dissolving 10 mg of standard quercetin in 10 mL of methanol (1000 μg/mL) and used as standard. The sample solution was prepared by extracting 2.0 g of dried powdered crude drug with 50 mL of methanol. The methanolic extract was filtered through the Whatman filter paper and evaporated to dryness under reduced pressure. The residue obtained was re-dissolved in 1.0 mL of methanol and used for chromatography.

#### HPTLC instrumentation and procedure

The sample was carefully spotted in the precoated silica gel aluminum plate 60 F-254 (10 cm × 10 cm with 0.2 mm thickness, E. Merck, Germany) using a Camag Linomat V (Switzerland) in the form of the bands of width 4.0 mm with a Camag microliter syringe with 150 nL/s constant application rate. A constant application rate 150 nL/s was employed. The slit dimension was kept at 4.0 mm × 0.45 mm and 20 mm/s scanning speed was employed. The mobile phase was composed of hexane:ethyl acetate: formic acid (5:4:1, v/v/v). The development of the HPTLC plate was carried out in ascending manner in twin trough glass chamber. The saturation time for the mobile phase 20 min in the saturation chamber and chromatogram was developed up tot the length 80 mm of the HPTLC plate and dried in the room temperature. The scanning was done in absorbance mode up to 570 nm.

### Animals

Healthy albino rats (Wistar strain) weight about 150-200 g were used. The entire animals used in the studies were kept in individual polyethylene cages and maintained standard condition (12 h dark and 12 h light circle; 25 ± 5°C; 40-60% humidity). The animals treated with standard fed *ad libitum* with normal laboratory chow standard pellet diet, purchased from the Hindustan Liver Limited, Mumbai, India. The animals were allowed to acclimate for 7 days before starting the experiments. All the studies were conducted in accordance with the Animal Ethical Committee as constituted by Siddhartha Institute of Pharmacy and the experimental protocol was approved by the Institutional Animal Ethical Committee of Siddhartha Institute of Pharmacy (1435/PO/a/11/CPCSEA).

The article "Paederia foetida Linn. leaf extract: an antihyperlipidemic, antihyperglycaemic and antioxidant activity" was retracted in 2025. Reasons: duplicated images; overlap with earlier publications; concerns about the images.

### Oral acute toxicity studies

For determination the oral acute toxicity studies the animals were starved overnight (16 h) and divided into six group (n = 6). Entire groups of tested animals received graded doses of *PF* extract dose raising level 100-2000 mg/kg body weight (i.e. 100, 250, 500, 1000, 2000 mg/kg body weight) and the animal was observed continuously for 2 h for on the basic of the following parameter after dosing [31,32]. The control group rats received vehicle only.

1: Behavioral changes viz., restlessness, irritability, alertness and fearfulness

2: Neurological changes viz., spontaneous activity, touch response, reactivity, pain response and gait

3: Autonomic changes viz., urination and defecation

These treatments observed for any changes and contraindication, death occurs during 24 h and 72 h.

### Effect of *PF* extract on glucose-hyperglycaemias animal model (glucose-loaded model, oral glucose tolerance test, OGTT)

This test was performed on overnight (16 h) famished normal albino wistar rat. The rats were randomly divided into seven groups and each group having 6 rats, while, [33].

Group I: rats was treated with vehicle only,

Group II: rats was treated with vehicle only + *PF* extract 500 mg/kg body weight,

Group III: rats was treated with vehicle only + Glucose 2 g/kg body weight,

Group IV: rats was treated with *PF* extract 100 mg/kg body weight,

Group V: rats was treated with *PF* extract 250 mg/kg body weight,

Group VI: rats was treated with *PF* extract 500 mg/kg body weight, and last group

Group VII: rats treated with Glibenclamide 10 mg/kg body weight.

After giving the respective option for the groups of the rats at mention above a single dose of 2 mg/kg of glucose was given to all the group after 30 min of initial feeding except group I and group II. Blood was drawn from the tail vein at regular intervals of time 0, 30, 60, 90, 120 and 150 min, blood glucose level were analyzed by the GOD-POD kit (Span diagnostic) following the given instruction by the manufacturer.

### Induction of diabetes

Swiss albino (wistar strain) rat was used for the induction of diabetes. Before the experimentation performs all animals were starving overnight (16 h). Diabetes was induced by single intraperitoneal injection (i.p.) of streptozotocin (60 mg/kg body weight) prepared by streptozotocin dissolving in 0.1 M citrate buffer (pH = 4. 5). All groups animal received the dose of STZ (60 mg/kg body weight) except normal control and normal control + *PF* (500 mg/kg) group rats. After 5 days all the groups’ animal blood samples collected from the puncturing the retro-orbits of the rat eyes and determine the blood glucose level using the GOD-POD method following the given instruction by the manufacture. The diabetes was confirmed by the elevating the blood glucose levels (220 mg/dl) were utilized for the study [34].

The article "Paederia foetida Linn. leaf extract: an antihyperlipidemic, antihyperglycaemic and antioxidant activity" was retracted in 2025. Reasons: duplicated images; overlap with earlier publications; concerns about the images.

### Experiment with design

After successfully developing the diabetes animals were divided into seven groups and each group contain six rats.

Group I: normal control rats administered vehicle only

Group II: normal control rats administered *PF* extract 500 mg/kg body weight

Group III: diabetic control rats administered drinking water alone

Group IV: tested rats administered *PF* extract 100 mg/kg body weight

Group V: tested rats administered *PF* extract 250 mg/kg body weight

Group VI: tested rats administered *PF* extract 500 mg/kg body weight

Group VII: tested rats administered glibenclamide 10 mg/kg body weight

All group rats received different doses of *PF* extract and glibenclamide using intragastric tube once daily for 28 days, continuously [35]. The blood samples of each animal were collected from the puncturing retro-orbital plexus and preserve anticoagulating agents; blood sample was centrifuged at 4000 RPM at 250°C for 15 min and analyzed for various biochemical parameters. The plasma insulin level was assayed by the radio-immunoassay method. All group rats serum glucose analysis was done by glucose oxidase-peroxidase (GOD-POD) method using Glucose estimation kit (Span Diagnostic, India). Other serum estimation done by spectrophotometrically using standard kit and following the given instruction. Serum triglyceride, total cholesterol, HDL (High Density Lipoprotein) cholesterol was analyzed by standard kits (Span Diagnostic, India) and other LDL (Low Density Lipoprotein) cholesterol [36], VLDL (Very Low Density Lipoprotein) were estimated with the help of the following formulas.

$$\mathrm{LDL}=\mathrm{TC}/1.19+\mathrm{TG}/1.9‒\mathrm{HDL}/1.1‒38\left(\mathrm{mg}/\mathrm{dL}\right)$$

$$\mathrm{VLDL}=\mathrm{triglycerides}\left(\mathrm{mg}/\mathrm{dL}\right)/5$$

### Estimation of antioxidant enzymes

For the estimation of the antioxidant enzymes, all groups rats’ liver successfully removed and homogenate. Liver homogenate prepared with ice chilled 10% potassium chloride solution, was used to measure the levels and activities of superoxide dismutase (SOD) [37], catalase (CAT) [38], glutathione peroxidase (GPx) and Malondialdehyde (MDA) by the method of [39,40].

The article "Paederia foetida Linn. leaf extract: an antihyperlipidemic, antihyperglycaemic and antioxidant activity" was retracted in 2025. Reasons: duplicated images; overlap with earlier publications; concerns about the images.

### Histopathology

At the end of the study 28 days all the groups animal were sacrificed under using mild anesthesia and isolated the different organ (heart, liver, pancreas and liver) of the animal for histopathology. All the animals were tested for absolute and relative organ weight and gross pathological lesions. The isolated organ (heart, liver, pancreas and liver) tissue fixed at 40% natural buffered formalin, dehydrated by passing through a graded series of alcohol, and embedded in paraffin blocks and 5 mm sections were developed using a semi-automated rotatory microtome. Hematoxylin and eosin were used for staining [40].

### Statistical analysis of experimental data

Values were presented as means ± standard error of the mean (S.E.M.). Statistical differences between the treatments and the controls were tested by one-way analysis of variance (ANOVA) followed by the Dennett’s test using the “Graph Pad Prism” statistic computer program. A difference in the mean values of p < 0.001 was considered to be statistically significant. Inhibition percentages were computed as follows:

$$\%\;\mathrm{inhibition}=\mathrm{Control}-\frac{\mathrm{test}}{\mathrm{control}}\times 100$$

## Result

### HPTLC analysis

The HPTLC finger print result for methanolic extract of *PF* showed the three phytoconstituents and corresponding the R_f_ values start from the 0.3 to 0.93 (Figure 1). The HPTLC analysis of *PF* extract showed the compound with R_f_ 0.77 as ascorbic acid as compared to the standard HPTLC graph of ascorbic acid (Figure 2).

**Figure 1:** **High performance thin liquid chromatography profiles of *Paederia foetida *** **extract.**

**Figure 2:** High performance thin liquid chromatography profiles of standard Ascorbic acid.

### Acute oral toxicity study in rats

Oral acute toxicity study, different doses of *PF* treated groups animals did not show any change in the behavioural, anatomical and neurological pattern. In complete study all the groups’ animals did not indicate any changes in the body weight and food consumption when compared to the vehicle treated groups. Therefore, it was concluded that the dose up to 2000 mg/kg of the *PF* extract was safe for the use.

### Effect of *PF* on oral glucose tolerance test

The consequence of the acute effect of graded doses of *PF* extract on blood sugar level of normal healthy rats and glucose loaded were presented in the Figure 3. Oral administration of different doses of *PF* extract and glibenclamide significantly decline (P < 0.001) the rise in blood glucose levels, after glucose administration. After loading the glucose, it was observed that glucose control group rats showed the higher AUC_glucose_ values (Figure 3). Oral administration of the different doses of the *PF* (100, 250 and 500 mg/kg) showed significantly (P < 0.001) lower AUC_glucose_ values as compared to the glucose control group rats (Table 1).

The article "Paederia foetida Linn. leaf extract: an antihyperlipidemic, antihyperglycaemic and antioxidant activity" was retracted in 2025. Reasons: duplicated images; overlap with earlier publications; concerns about the images.

**Figure 3:** **Oral glucose tolerance and AUC of *PF *leaves extracts in normal rats.** Values are given as mean ± S.E.M. of six rats in each group. *p ≤ 0.05, **p ≤ 0.005, ***p ≤ 0.001 compared with normal control values.

**Table 1:** **Pharmacokinetic parameters of *Paederia foetida *** **Linn. extract in Oral glucose tolerance test**

**S. No**		**Pharmacokinetic parameters**		
		**C**_**max **_**(mg/dl)**	**t**_**max **_**(min)**	**AUC (mg.min/dl)**
**1**	**Glucose control**	119.4	30	16239
**2**	**Glucose +** ***PF *** **I (100 mg/kg)**	114.2	30	14847
**3**	**Glucose +** ***PF *** **II (250 mg/kg)**	110.2	30	13929
**4**	**Glucose +** ***PF *** **III (500 mg/kg)**	105.2	30	12645
**5**	**Glucose + Glibenclamide (10 mg/kg)**	107	30	13020

Each parameter represents the mean of Six animals. Area under curve (AUC) values. t_max_, time at maximum observed concentration; C_max_, maximum concentration.

### Effect of *PF* on blood glucose level

The antidiabetic effect of repeated oral administration of *PF* leaves extract on STZ (streptozotocin) induced diabetic rats was presented in Table 2. Three different doses of *PF* leaves extract (100, 250 and 500 mg/kg) to STZ induced diabetic rats caused significantly (P < 0.001) decline the blood glucose level which was showing dose and duration of treatment. Maximum reduction of blood glucose was observed at day 28 (55.74%, 61.76% and 69.12% respectively). *PF* dose 500 mg/kg shown the maximum reduction of the high blood glucose level when compared to the two other different grades of doses of *PF*. On the other hand glibenclamide show the decreased level of blood glucose 65.27.

**Table 2:** **Effect of *Paederia foetida *** **Linn. on biochemical parameters in STZ-induced diabetic rats**

**S. No.**	**Biochemical parameter**	**Normal control**	**Normal control + PF (500 mg/kg)**	**STZ-Diabetic control**	**STZ diabetes + PF I (100 mg/kg)**	**STZ diabetes + PF II (250 mg/kg)**	**STZ diabetes + PF III (500 mg/kg)**	**STZ diabetes + Glibenclamide (10 mg/kg)**
**1**	**Fasting plasma glucose (mg/dL)**	81.8 ± 0.201	79.8 ± 0.245	348.4 ± 2.781^a^	154.2 ± 1.812^b^	133.2 ± 0.861^b^	107.6 ± 1.749^b^	122 ± 1.844^b^
**2**	**Fasting Plasma Insulin (μU/mL)**	11.4 ± 0.509	11.4 ± 0.245	2.4 ± 0.453^**a**^	4.2 ± 0.373^**b**^	6.2 ± 0.374^**b**^	10.6 ± 0.438^**b**^	9.6 ± 0.123^**b**^
**3**	**Glycated Heamoglobin (A1c) (%)**	1.24 ± 0.092	1.24 ± 0.0812	4.86 ± 0.178^**a**^	3.96 ± 0.238^**b**^	2.82 ± 0.861^**b**^	1.52 ± 0.0431^**b**^	1.86 ± 0.093^**b**^
**4**	**Hexokinase (μg/mg of tissue)**	151 ± 3.24	150.6 ± 3.108	88.4 ± 1.806^**a**^	115.2 ± 1.497^**b**^	131 ± 1.643^**b**^	147.2 ± 1.281^**b**^	141.6 ± 2.088^**b**^
**5**	**Glucose-6-Phosphatase (unit/mg of tissue)**	8 ± 0.707	8 ± 0.717	14.4 ± 0.927^**a**^	13.4 ± 0.509^**b**^	11.4 ± 0.432^**b**^	8.4 ± 0.436^**b**^	9.8 ± 0.374^**b**^
**6**	**Fructose-1-6-biphosphatase (unit/mg of tissue)**	26.8 ± 1.241	27 ± 1.517	54.8 ± 1.281^**a**^	43 ± 1.871^**b**^	38.2 ± 1.497^**b**^	30 ± 0.707^**b**^	31 ± 0.431^**b**^
**7**	**Total Cholesterol (mg/dL)**	66.2 ± 1.715	66.8 ± 1.393	141.2 ± 2.634^**a**^	129.8 ± 1.53^**b**^	101.8 ± 1.934^**b**^	76.2 ± 2.01^**b**^	84 ± 2.302^**b**^
**8**	**Triglycerides (mg/dL)**	78 ± 1.975	78.2 ± 1.431	144.8 ± 3.04^**a**^	131 ± 1.789^**b**^	110.2 ± 1.828^**b**^	91 ± 1.703^**b**^	98 ± 1.265^**b**^
**9**	**Total HDL Cholesterol (mg/dL)**	57 ± 1.14	57 ± 0.124	25.4 ± 1.208^**a**^	39 ± 1.225^**b**^	44.4 ± 1.03^**b**^	51.6 ± 0.927^**b**^	53.4 ± 0.927^**b**^
**10**	**Total LDL Cholesterol (mg/dL)**	6.4 ± 0.18	6.8 ± 0.431	86.8 ± 0.818^**a**^	64.6 ± 0.053^**b**^	35.4 ± 0.538^**b**^	8.4 ± 1.121^**b**^	11 ± 0.742^**b**^
**11**	**Total VLDL Cholesterol (mg/dL)**	15.6 ± 0.295	15.72 ± 0.132	28.96 ± 0.608^**a**^	26.2 ± 0.375^**b**^	22 ± 0.365^**b**^	18.2 ± 0.253^**b**^	10.6 ± 0.341^**b**^

Values are given as mean ± S.E.M. of six rats in each group. ^a^(*P* <0.01) compared with the corresponding value for normal control animals (group I); ^b^(*P* <0.01) compared with the corresponding value for diabetic control animals (group III); ns-non significant.

The article "Paederia foetida Linn. leaf extract: an antihyperlipidemic, antihyperglycaemic and antioxidant activity" was retracted in 2025. Reasons: duplicated images; overlap with earlier publications; concerns about the images.

### Effect of *PF* of plasma insulin

STZ treated group rat significantly decrease in serum insulin as compared to the normal control groups rat. Normal control rat received a *PF* dose (500 mg/kg) shown slightly improved the plasma insulin level as compared to the normal control group rat. STZ induced diabetic rat treated with different doses of *PF* significantly improved the plasma insulin level as compared to the diabetic control group rat (Table 2). On the all three graded doses, 500 mg/kg showed most significant improvement in decreasing the insulin level as compared to the diabetic control group rats.

### Effect of *PF* on glycated haemoglobin (A1c)

Oral administration of different doses of *PF* was significantly decreased the level of glycated haemoglobin (A1c) in STZ-induced treated diabetic rats (Table 2). The level of glycated haemoglobin was normal in the wistar rats fed with normal diet (group I) in conjunction with the normal control rats received *PF* with a dose of 500 mg/kg (group II). STZ induced diabetic rat showed a marked increase in the level of glycated haemoglobin (A1c) in STZ-induced treated diabetic rats. Upon the oral administration of the different doses of *PF* and glibenclamide significantly decrease the level of glycated haemoglobin as compared to the diabetic control.

### Effect of *PF* on hexokinase

Hexokinase level was observed a decline in STZ treated group rat as compared to the normal control group (Table 2). Administration of *PF* dose 500 mg/kg in the normal rat showed little or no changes in the level of hexokinase. STZ induced diabetic rat treated with different doses of *PF* showed significant improvement in the degree of hepatic hexokinase. STZ induced diabetic rat treated with *PF* dose 500 mg/kg showed maximum improvement in the level of hexokinase as compared to the other graded dose and glibenclamide treated group rat.

### Effect of *PF* on glucose-6-phosphate

It is the evident from the table that upon oral administration of STZ to wistar rats showed the increased level of glucose-6-phosphatase (Table 2). Oral administration of the *PF* dose 500 mg/kg did not show any change in the level of glucose-6-phosphatase. When STZ induced diabetic rat treated with different doses of *PF,* there was a significant (P < 0.001) decreased the level of glucose-6-phosphatase in dose dependent manner. Upon administration of different doses of *PF* and Glibenclamide, significant (P < 0.001) decline in the level of glucose-6-phosphatase has been observed but the dose *PF* 500 mg/kg was found to be more effective to decline the high level of glucose-6-phosphatase.

### Effect of *PF* on fructose-1-6-biphosphatase

The oral administration of *PF* dose 500 mg/kg has shown the equal level of fructose-1-6-biphosphatase compared to the normal control group rats. STZ induced diabetic rats significantly (P < 0.001) improved the level of fructose-1-6-biphosphatase as compared to the normal control group rat (Table 2). Upon oral administration of different doses of *PF* leaves extract and glibenclamide significantly (P < 0.001) decline the level of the fructose-1-6-biphosphatase. The *PF* dose 500 mg/kg showed the higher decline capability of fructose-1-6-biphosphatase as compared to the other dose of the *PF* and glibenclamide.

### Effect of *PF* on lipid profile

Effect of different doses of *PF* leaves extract on lipid profile level was evaluated. The level of cholesterol, triglyceride, LDL (low density cholesterol) and VLDL (very low density cholesterol) were increased and the level of HDL (high density cholesterol) was decreased in the STZ induced diabetic rat as compared to the normal control group rats. The oral administration of *PF* dose 500 mg/kg to the normal rat did not show any change in the lipid profile (Table 2). Oral administration of different doses (100 mg/kg, 250 mg/kg and 500 mg/kg, p.o.) of *PF* were showed percentage reduction in cholesterol (14.80%, 22.90%, 32.82%), triglyceride (11.48%, 21.07%, 33.72%), LDL (26.82%, 44.18%, 65.08%) and VLDL (11.48%, 21.07%, 33.72%), compared to the diabetic control rat group and the level of HDL (29.93%, 49.64%, 69.34%), was increased when compared to the diabetic control rat. Oral administration of *PF* dose 500 mg/kg showed the maximum benefit as compared to the other dose of the *PF* and glibenclamide in reducing the level of cholesterol, triglyceride, LDL cholesterol and VLDL cholesterol and increasing the level of HDL cholesterol as compared to the STZ induced diabetic control rat.

The article "Paederia foetida Linn. leaf extract: an antihyperlipidemic, antihyperglycaemic and antioxidant activity" was retracted in 2025. Reasons: duplicated images; overlap with earlier publications; concerns about the images.

### Changes in body weight

STZ treated diabetic rats showed significant loss the body weight as compared to the normal control group rat (Table 2). STZ treated diabetic control group rat significantly reduced the body weight as compared to the normal control group rats. STZ induced diabetic rat treated with different doses of *PF* (100 mg/kg, 250 mg/kg and 500 mg/kg) and glibenclamide (10 mg/kg) exhibited significant (P < 0.001) improvement in the body weight as compared to the diabetic control group rats.

### Effect of *PF* on antioxidant enzymes

Table 3 represents the activity of the antioxidant enzyme like SOD, CAT, GPx and MDA in the normal and diabetic rat. The level of SOD, CAT, GPx decreased and MDA level increased in the STZ induced diabetic group rat (Table 3). Upon administration of *PF* with dose 500 mg/kg in the normal control group rat did not indicate any alteration in the level of antioxidant enzymes. Oral administration of different doses of *PF* (100 mg/kg, 250 mg/kg and 500 mg/kg) significantly improved the level of SOD, CAT, GPx and decline the level of MDA as compared to the normal control group rats. Oral administration of *PF* doses (100 mg/kg, 250 mg/kg and 500 mg/kg) brought to the value to near the normal, similar to the glibenclamide treated group rats.

**Table 3:** **Effect of *Paederia foetida *** **Linn. on antioxidant marker in STZ-induced diabetic rats**

**S. No.**	**Biochemical parameter**	**Normal control**	**Normal control + PF (500 mg/kg)**	**STZ-Diabetic control**	**STZ diabetes + PF I (100 mg/kg)**	**STZ diabetes + PF II (250 mg/kg)**	**STZ diabetes + PF III (500 mg/kg)**	**STZ diabetes + Glibenclamide (10 mg/kg)**
**1**	**SOD (U/mg of protein)**	7.8 ± 0.374	7.6 ± 0.245	2.2 ± .374^**a**^	4.2 ± 0.374^**b**^	5.2 ± 0.374^**b**^	7 ± 0.316^**b**^	6.6 ± 0.245^**b**^
**2**	**CAT (U/mg of protein)**	72 ± 1.612	70.6 ± 1.72	38 ± 1.732^**a**^	45.8 ± 1.068^**b**^	53.8 ± 1.158^**b**^	68 ± 1^**b**^	65.4 ± 1.077^**b**^
**3**	**GPx (nmole/mg of protein)**	32.8 ± 1.02	32.6 ± 1.208	13.2 ± 0.374^**a**^	19 ± 0.707^**b**^	24.6 ± 0.509^**b**^	31 ± 0.458^**b**^	29.6 ± 0.927^**b**^
**4**	**MDA (nmole/mg of protein)**	0.2 ± 0.011	0.21 ± 0.007	0.54 ± 0.013^**a**^	0.39 ± 0.009^**b**^	0.32 ± 0.005^**b**^	0.25 ± 0.005^**b**^	0.26 ± 0.003^**b**^

Values are given as mean ± S.E.M. of six rats in each group. ^a^(*P* <0.01) compared with the corresponding value for normal control animals (group I); ^b^(*P* <0.01) compared with the corresponding value for diabetic control animals (group III); ns-non significant.

The article "Paederia foetida Linn. leaf extract: an antihyperlipidemic, antihyperglycaemic and antioxidant activity" was retracted in 2025. Reasons: duplicated images; overlap with earlier publications; concerns about the images.

### Effect of *PF* on liver

STZ induced diabetic rat liver histopathology has shown the accumulation of fat droplet and large area of hepatocytes as compared to the histopathology of the normal control group rat liver histopathology. Oral administration of different doses of *PF* group rat showed the improved liver histopathology as compared to the diabetic control group rats (Figure 4). STZ induced diabetic rat treated with *PF* dose 100 mg/kg depicted the fat droplet accumulation in the liver as compared to the normal control groups rat but less than the diabetic control group rats. Other graded dose of *PF* 250 mg/kg showed the improved effect on the liver histopathology on the accumulation of the fat droplet as compared to the *PF* dose 100 mg/kg and diabetic control group rat. *PF* dose 500 mg/kg showed the systematic effect and did not show the any droplet of the fat accumulation on the liver histopathology as compared to the diabetic control. Glibenclamide treated group rat shown the liver histopathology similar to the normal control group rats (Figure 5).

**Figure 4:** ***Paederia Foetida *Linn. leaves extract effect on liver histopathology in normal and STZ induced diabetic rats. (A)** Normal control: Histopathology of normal control rat did not display any sign of the changes **(B)** Diabetic control: Yellow arrow display the deposition of the fat micro and macro droplet. **(C)***PF* I (100 mg/kg): STZ induced diabetic rat display the micro droplet deposition on the liver histopathology (Yellow arrow) **(D)***PF* II (250 mg/kg): *PF* increasing dose display the few micro droplet deposition of the fats (Yellow arrow) **(E)***PF* III (500 mg/kg): *PF* dose 500 mg/kg did not display any change or absorbent. **(F)** Glibenclamide (10 mg/kg): Glibenclamide treated group rat display the normal histopathology. The samples were obtained from the same liver anatomical regions. For each group, 6 rats were examined and 80 pictures were taken. The above picture for each group was chosen randomly from the 50 pictures in this group. Original magnification, 10×.

The article "Paederia foetida Linn. leaf extract: an antihyperlipidemic, antihyperglycaemic and antioxidant activity" was retracted in 2025. Reasons: duplicated images; overlap with earlier publications; concerns about the images.

**Figure 5:** ***Paederia Foetida *Linn. leaves extract effect on liver histopathology in normal and STZ induced diabetic rats. (A)** Normal control: Normal control group did not display any changes **(B)** Diabetic control: Display the fat deposition (Yellow arrow) **(C)***PF* I (100 mg/kg): Histopathology display the some pat having the micro droplet of fat deposition (Yellow arrow) **(D)***PF* II (250 mg/kg): *PF* treated drug displaying the fat deposition (Yellow arrow) **(E)***PF* III (500 mg/kg): *PF* treated group did not display the any changes and fat deposition of the liver histopathology **(F)** Glibenclamide (10 mg/kg): Glibenclamide treated group did not display any changes, histopathology similar to the normal control group. The samples were obtained from the same liver anatomical regions. For each group, 6 rats were examined and 50 pictures were taken. Original magnification, 40×.

### Effect of *PF* on heart

STZ induced diabetic group rat disturbed the lipid profile and showed direct effect on the heart. Histopathology of heart showed the distorted intercalated discs and interstitial spaces, in STZ induced diabetic group rats (Figure 6). Now, the treatment with different doses of *PF* and glibenclamide showed the systematic effect on the heart histopathology. The distortion of intercalated discs was decline at dose dependent manner. The dose *PF* 500 mg/kg shown the histopathology of the heart almost similar to the normal heart. Glibenclamide treated group rat shown the histopathology similar to the normal control group rats (Figure 7).

**Figure 6:** ***Paederia Foetida *Linn. leaves extract effect on heart histopathology in normal and STZ induced diabetic rats. (A)** Normal control: Normal histopathology **(B)** Diabetic control: Display increased interstitial space and distort the intercalated disc (yellow arrow). **(C)***PF* I (100 mg/kg): Display less interstitial space and intercalated disc (yellow arrow). **(D)***PF* II (250 mg/kg): *PF* treated drug display only space in intercalated disc (yellow arrow). **(E)***PF* III (500 mg/kg): Did not display any changes of the heart histopathology **(F)** Glibenclamide (10 mg/kg): Histopathology similar to the normal group. The samples were obtained from the same liver anatomical regions. For each group, 6 rats were examined and 50 pictures were taken. Original magnification, 10×.

The article "Paederia foetida Linn. leaf extract: an antihyperlipidemic, antihyperglycaemic and antioxidant activity" was retracted in 2025. Reasons: duplicated images; overlap with earlier publications; concerns about the images.

**Figure 7:** ***Paederia Foetida *Linn. leaves extract effect on heart histopathology in normal and STZ induced diabetic rats. (A)** Normal control: Did not display any changes **(B)** Diabetic control: Histopathology of diabetic control group rat display increased interstitial space and distort the intercalated disc (yellow arrow) **(C)***PF* I (100 mg/kg): Histopathology of tested drug display decreased interstitial space and intercalated disc (yellow arrow) **(D)***PF* II (250 mg/kg): Display only interstitial space (yellow arrow) **(E)***PF* III (500 mg/kg): Display some intercalated disc (Yellow arrow) **(F)** Glibenclamide (10 mg/kg): Similar display live the normal control group histopathology. The samples were obtained from the same liver anatomical regions. For each group, 6 rats were examined and 50 pictures were taken. Original magnification, 40×.

### Effect of *PF* on kidney

Histopathology of kidney was determined after 28 days treatment of different doses of *PF* and glibenclamide in STZ induced diabetic rats. Normal control group rat kidney histopathology showed the normal size of the bowman capsule and glomerulus. STZ induced diabetes rats’ kidney histopathology depicted the inflamed blood vessels, fat deposition, increase in the thickness of bowman capsules and change in size of the glomerulus. Oral administration of different doses of *PF* reduced the inflammatory blood vessels. The treatment with *PF* 100 mg/kg dose showed the reduction of the inflammatory blood vessels and slightly shorter bowman capsules and glomerulus as compared to the diabetic control group rat kidney histopathology (Figure 8). Other *PF* dose 250 mg/kg kidney histopathology have shown the disappearance of the inflamed blood vessels and depicted the smaller size of the bowman capsules and glomerulus. *PF* dose 500 mg/kg caused complete disappearance of the inflamed blood vessel, but bowman capsule shown to be slightly bigger as compared to the normal control group rats. Glibenclamide treated group rat kidney histopathology did not show the any inflamed blood vessels and exhibiting the bowman capsules similar to the normal control group rat histopathology (Figure 9).

**Figure 8:** ***Paederia Foetida *Linn. leaves extract effect on kidney histopathology in normal and STZ induced diabetic rats. (A)** Normal control: Normal control group rat histopathology shown normal size of glomerulus and bowman capsule (Green arrow) **(B)** Diabetic control: Diabetic control group rat histopathology display the inflamed blood vessels (Red arrow), bigger size of bowman capsule, glomerulus and fat deposition (Yellow arrow) **(C)***PF* I (100 mg/kg): *PF* tested drug histopathology display the inflammation in blood vessels (brown arrow), bigger size bowman capsule and fat deposition (yellow arrow) **(D)***PF* II (250 mg/kg): *PF* treated drug group rat histopathology display fat deposition (yellow arrow) and inflammatory blood cells (Red arrow). **(E)***PF* III (500 mg/kg): *PF* treated group display the normal histopathology only increase the size of bowman capsule (green arrow). **(F)** Glibenclamide (10 mg/kg): Histopathology of glibenclamide treated group rat display the normal kidney but bowman capsule bigger in size (Green arrow). The samples were obtained from the same liver anatomical regions. For each group, 6 rats were examined and 50 pictures were taken. Original magnification, 10×.

The article "Paederia foetida Linn. leaf extract: an antihyperlipidemic, antihyperglycaemic and antioxidant activity" was retracted in 2025. Reasons: duplicated images; overlap with earlier publications; concerns about the images.

**Figure 9:** ***Paederia Foetida *Linn. leaves extract effect on kidney histopathology in normal and STZ induced diabetic rats. (A)** Normal control: Bowman capsule in average size **(B)** Diabetic control: Diabetic control group rat histopathology display inflammatory cells in blood vessels (Red arrow) and fat deposition (Yellow arrow). **(C)***PF* I (100 mg/kg): *PF* treated group display inflammatory cell in blood vessels (Red arrow) and deposition of fat (Yellow arrow). **(D)***PF* II (250 mg/kg): *PF* tested drug group histopathology few parts display the fat deposition (Yellow arrow) and inflamed cells in blood vessels (Red arrow). **(E)***PF* III (500 mg/kg): *PF* treated drug display the normal histopathology few changes in the size of bowman capsules. **(F)** Glibenclamide (10 mg/kg): Glibenclamide treated group rat did not display any changes in the histopathology, only bigger size of bowman capsules. The samples were obtained from the same liver anatomical regions. For each group, 6 rats were examined and 80 pictures were taken. Original magnification, 40×.

### Effect of *PF* on pancreas

Histopathology studies of the experimental rat were measured after 28 days continuous administration of different doses of *PF* and glibenclamide. STZ induced diabetic rat had shown the reduction of the isles of the Langerhans, reduced size of β cells and extensive necrosis changes followed by fibrosis and atrophy. Histopathology studies of pancreas of STZ induced diabetic rat displayed reduction of the islets of Langerhans, damaged or reduced size of β cells and extensive necrosis changes followed by fibrosis and atrophy (Figure 10). STZ induced diabetic rat treated with different doses of *PF* (100 mg/kg, 250 mg/kg, and 500 mg/kg) and glibenclamide restored the necrotic and fibrotic changes and raised the number of β cells (Figure 11).

**Figure 10:** ***Paederia Foetida *Linn. leaves extract effect on pancreas histopathology in normal and STZ induced diabetic rats. (A)** Normal control: Normal control group rat histopathology display the normal size of islet of langerhans (Green arrow) **(B)** Diabetic control: Diabetic control histopathology display the focal necrosis (yellow arrow) and bigger in the size of islets of langerhans (Black arrow). **(C)***PF* I (100 mg/kg): *PF* tested drug display bigger size of islet (Black arrow) and focal necrosis (Yellow arrow). **(D)***PF* II (250 mg/kg): *PF* tested drug display only focal necrosis (Yellow arrow) **(E)***PF* III (500 mg/kg): *PF* tested drug display normal size of islet (Green arrow) **(F)** Glibenclamide (10 mg/kg): Glibenclamide treated rat pancreas showing normal islet (Green arrow). For each group 6 rats were examined and 50 pictures were taken. Original magnification, 10×.

The article "Paederia foetida Linn. leaf extract: an antihyperlipidemic, antihyperglycaemic and antioxidant activity" was retracted in 2025. Reasons: duplicated images; overlap with earlier publications; concerns about the images.

**Figure 11:** ***Paederia Foetida *Linn. leaves extract effect on pancreas histopathology in normal and STZ induced diabetic rats. (A)** Normal control: Normal control group display the normal islet (Red arrow) **(B)** Diabetic control: Diabetic control rat histopathology display the islet enlargement (Blue arrow) and focal necrosis (Yellow arrow) **(C)***PF* I (100 mg/kg): *PF* tested drug histopathology display bigger size of islet (Blue arrow) and focal necrosis (Yellow arrow) **(D)***PF* II (250 mg/kg): Other *PF* tested drug display focal necrosis (Yellow arrow) and islet enlargement (Blue arrow). **(E)***PF* III (500 mg/kg): *PF* tested drug display normal size of islet (Red arrow) **(F)** Glibenclamide (10 mg/kg): Glibenclamide treated group rat histopathology display normal islet (Red arrow) similar to the normal control group. For each group 6 rats were examined and 50 pictures were taken. Original magnification, 40×.

## Discussion

The present investigation study discusses about the antidiabetic, antihyperlipidemic and antioxidant potential effect of the methanolic leaf extract of *Paederia foetida* Linn. in normal and streptozotocin induced diabetic rats. Phytochemical screening shows that the *Paederia foetida* Linn. Leaves extract consists the richest source of the various bioactive compounds. Acute toxicity studies of the *Paederia foetida* Linn. leaf extract reveals the non toxic nature of the extract at the dose upto 2000 mg/kg, there was no lethality or any other toxic reactions found with the selected dose until the conclusion of the study.

In the present study, STZ has been used as a diabetogenic agent to induce the diabetes in rodents. Low dose of STZ has been commonly used for the induction of type I diabetes (Insulin dependent diabetes mellitus). After treatment with low dose of STZ survival and regeneration of pancreatic β-cells is possible in type I diabetes [41]. Streptozotocin (2-deoxy-2-(N-methyl-N-nitrsourea) -1-D-glucopyranose) is a nitrosourea compound obtained from the soil microbe *Streptomyces achromogenes*[42]*,* which is the potent alkylating agent that exerts its effect on the pancreatic β-cells via glucose transporter-GLUT2, causing induction of methylation of DNA and results in damage of DNA. Damaged DNA, activate the poly (ADP-Ribose) polymerase, leading to NAD^+^ depletion in pancreatic β-cells [43]. STZ also acts as a nitric oxide donor in pancreatic islets, enhances O_2_^-^ radical fragmentation in islet cells. As a result, pancreatic β-cell death occurred by apoptosis and necrosis ensued, which in turn decreases proinsulin synthesis [44].

The article "Paederia foetida Linn. leaf extract: an antihyperlipidemic, antihyperglycaemic and antioxidant activity" was retracted in 2025. Reasons: duplicated images; overlap with earlier publications; concerns about the images.

A lot of conventional drugs available in the market to cure and maintain the blood glucose level in diabetic patients. But most of the time sulfonylurea, such as glibenclamide has been used as a standard antidiabetic drug to compare the efficacy of a variety of antihyperglycemic compounds. Glibenclamide exerts their anti-diabetic action by stimulating insulin secretion. In our study, we have compared our plant based drug with the standard drug, Glibenclamide [45].

In the treatment of diabetes, there is a limited availability of the oral pharmacological agents. Now the current researches focus on the discovery of the novel oral pharmacological agents to control of blood glucose, hyperlipidemic and antioxidant with different mechanism of action. Allopathic medicines are widely available in the market to cure the diabetes but they are associated with the limitation due to their specific action and side effect. The best alternate to cure the diabetes is the alternative system of medicine which has a very long history. Plant derived antidiabetic agents are gaining popularity day by day at around the world for its effectiveness antidiabetic activity and minimal side effects [46].

In the subject field of the normolglycemic rats, *PF* showed the hypoglycaemic effect at dose dependent manner. In the study of the oral glucose tolerance test result showed the better utilization of the glucose by the animals. This plausible outcome that the different doses of the *PF* extract has the sound capacity to block glucose absorption. In the OGTT studies [34], it could be concluded that *PF* dose 500 mg/kg showed the maximum improvement in the glucose tolerance as compared to the other dose of *PF* and glibenclamide.

STZ induced diabetic rat increased the blood glucose level and decrease the insulin level due to STZ induced abnormalities in the β cell function [47]. The outcome of the case indicates that the methanolic leaf extract of *PF* restrained the blood sugar level in normoglycaemic, glucose-hypoglycaemic and STZ induced diabetic rats. In normoglycemic and STZ induced diabetic rats hypoglycaemic action of the *PF* leaf extract was observed at dose manner, with prolonged hypoglycaemic effect at higher dose. The *PF* dose, 500 mg/kg, is most effective to diminish the raised blood glucose level. The *PF* dose had shown the best result when compared to the synthetic drug glibenclamide (Table 2). The possible mechanism of activity of *PF* leaves extract may be stimulating the insulin secretion and regeneration of the β-cells of the pancreas or increasing cellularity of the islet tissue and regeneration of the granules in the β-cells. Based upon the result it can be hypothesized that *PF* declined the level of the blood glucose and improved the pancreas insulin level [45]. This hypothesis has been further confirmed by the histopathology studies of the pancreas which showed protection of the pancreas from the toxic effect of microbial streptozotocin (Figures 10 and 11). The leaf extract has shown the similar mechanism of action as glibenclamide, i.e. stimulating the insulin secretion.

The article "Paederia foetida Linn. leaf extract: an antihyperlipidemic, antihyperglycaemic and antioxidant activity" was retracted in 2025. Reasons: duplicated images; overlap with earlier publications; concerns about the images.

In the STZ induced diabetes rats, reduced body weight was continuously observed. Body weight was continuously decreasing in the STZ induced diabetic rat due to muscle destruction or degeneration of structural proteins [48]. Normal rat and STZ induced diabetic rat treated with different doses of the *PF* leaves extract and glibenclamide, revealed body weight gain as compared to the diabetic control group rats. The result suggests that the different doses of the *PF* and glibenclamide shown the protective effect in the regulation of the muscle wasting (reversal of gluconeogenesis). Normal control group rat treated with *PF* dose, 500 mg/kg, has shown the better improvement in the body weight as compared to the diabetic control and normal control group rats (Table 2).

In normal condition, glycated hemoglobin make 3.4-5.8% of total hemoglobin and a small portion of blood glucose, usually 4.5-6%, has been covalently bonded to the red blood cells in hemoglobin. In diabetic condition increased level of the glycated hemoglobin due to increased level of blood glucose, which has been added to the N terminus of hemoglobin and producing the increased level of glycated hemoglobin [49]. In STZ induced diabetic condition glycated heamoglobin has been increased four times more than the normal level. Our result lie in agreement with this well known fact that treatment with *PF* for 28 days decreased the excess level of the glycated hemoglobin (Table 2), which indicates the improved echelon of glycemic control.

The article "Paederia foetida Linn. leaf extract: an antihyperlipidemic, antihyperglycaemic and antioxidant activity" was retracted in 2025. Reasons: duplicated images; overlap with earlier publications; concerns about the images.

Some of the researcher claims that the oxidative stress plays an important role in the microvascular and macrovascular complication of diabetes [50]. In diabetes condition organ damage is the most common problem due to the defective cell antioxidant response against the oxidative stress generated in the diabetic condition [51]. Oxygen free radical plays an important role in the production of the oxidative stress. The free radical reacts with all biological substance, mainly polyunsaturated fatty acids and this reaction will lead to the cell membrane constituents lead to the lipid peroxidation [52]. During oxidative stress increased production of Lipid peroxidation impairs the membrane function by decreasing membrane fluidity and changing the activity of membrane-bound enzyme and receptors [53]. These findings suggest that antioxidant treatment may be beneficial for diabetic patients. STZ induced diabetic rat increased the level of the antioxidant marker, several mechanisms of action are involved like overproduction of the free radical, glucose autooxidation, protein glycation, formation of advanced glycation products and polyol pathway [54]. In STZ induced diabetic condition increased level of the hepatic and renal MDA (as an indicator of the Lipid peroxidation) level and decreasing SOD, CAT, GPx level indicates the increased free radical generation. STZ induced diabetic rat treated with different doses of *PF* leaf extract decreased the level of MDA and improved the level of SOD, CAT and GPx. SOD is an important defense enzymatic antioxidant, the principal activity of the SOD is scavenge superoxide radical (O_2_^-^) from to hydrogen peroxide (H_2_O_2_) and secondary action diminishes the toxic effects caused by the free radical reaction. The other enzymatic antioxidant CAT is a hemoprotein, which cause reduction of the hydrogen peroxide and known to be involved in the detoxification of hydrogen peroxide concentration [55]. The other antioxidant glutathione peroxidase has been able to reduce lipid hydroperoxidase and hydrogen peroxide level. STZ induced diabetic rat with higher level of blood glucose can inactivate the SOD, CAT and GPx by fluctuating these proteins thus producing induced oxidative stress, which is turn, cause lipid peroxidation [56]. STZ induced diabetic rat treated with different doses of *PF* leaves extract brought back the level of SOD, CAT and GPx activities near to normal control group rat indicating the usefulness of *PF* in attenuating the oxidative stress in diabetic liver.

In the diabetes condition hypertriglyceridemia and hypercholestermia are the common factors involved in the development of the atherosclerosis and coronary heart disease. This occurs due to lack of the insulin, which activates the lipase enzyme, hydrolyzed triglyceride (TG) and releasing the fatty acid and glycerol into the circulating blood. The level of the triglyceride has been increased in the STZ induced diabetic rat due to decreased level of insulin, which causes failure to the activate lipoprotein lipase thereby causing hypertriglyceridemia [57]. STZ induced diabetes often involves abnormal lipid metabolism which is a metabolic disorder in diabetes complications [58]. In diabetes, increased level of total cholesterol, is one of the major factors for coronary heart disease (hyperlipidaemia) and its incidence of atherosclerosis. In our studies STZ induced diabetic rats have shown increased level of the total cholesterol. Treatment with the different doses of *PF* declines the highest level of total cholesterol and brought back the normal control level. The exact mode of action is unknown which involves the decline of total cholesterol. Decline in the cholesterol level achieved by the *PF* leaf extract has been shown to have direct effect on lipids or controlling the blood glucose level. LDL (Low density lipoprotein) and VLDL (Very low density lipoprotein) start depositing in the peripheral tissue in the diabetic condition [45]. STZ induced diabetic rat increased the level of LDL and VLDL. The treatment has been started with different doses of *PF* leaf extract produces a decline in the higher level of LDL and VLDL cholesterol. On the other hand HDL (High density lipoprotein) cholesterol has been shown to decrease in the diabetic condition. Treatment with *PF* leaf extract for 28 days produces diminished level of TC, TG, LDL, and VLDL while the level of HDL Cholesterol has been significantly reduced [34]. These data suggest that the *PF* leaf extract possesses the excellent ability to ameliorate the lipid profile on the diabetic rats.

The article "Paederia foetida Linn. leaf extract: an antihyperlipidemic, antihyperglycaemic and antioxidant activity" was retracted in 2025. Reasons: duplicated images; overlap with earlier publications; concerns about the images.

The liver plays an important role in the regulation of glucose metabolizing enzyme. Its regulate glucose-6-phosphatase, hexokinase and fructose-1-6-biphosphate. STZ induced diabetic rats have increased the level of glucose-6-phosphatase, which in turn enhance the production of fats from the carbohydrates results in increased level deposition of fats in the liver and kidney [59]. The deposition of the fats in the kidney and liver has been supported by the histopathological study. STZ induced diabetic rat treated with different doses of *PF* significantly decreased the level of glucose-6-phosphatase. Histopathological studies also supported the systematic effect of the *PF* extract at dose dependent manner. Fructose-1-6-biphosphateis the other vital enzyme convert glucose into energy and plays an important role in the glycolysis [60,61]. STZ induced diabetic rats has been shown to have increased level of fructose-1-6-biphosphate. Treatment with *PF* leaves extract causes sharp decline in the higher level of fructose-1-6-biphosphate. Other liver enzyme hexokinase take part in the conversion of glucose into glucose-6-phosphatase and utilization of the glucose into the energy [62-65]. In STZ induced diabetic rats the collapse in glucose metabolism, disturb the capacity of the liver to synthesize glycogen, decline the level of hexokinase and decreased the use of energy. STZ induced diabetic rat treated with different doses of the *PF* leaf extract improved the level of hexokinase at dose dependent manner (Table 2).

## Conclusion

In conclusion, our investigation has clearly indicated that the leaf extract of *Paederia foetida* Linn. showed remarkable antihyperglycemic activity due to its possible systematic effect involved in the pancreatic and extra pancreatic mechanism. Furthermore, the antihyperlipidemic activity was exerted by lowering the higher level of lipid profile and decreasing the intercalated disc space in the heart. The antioxidant activity of extract was due to inhibition of lipid peroxidation and improved level of SOD, GPx and CAT. It was corroborateral that the extract of the Paederia *foetida* Linn leaves exhibited significant antidiabetic, antihyperlipidemic and antioxidant potential.

## Competing interests

The authors declare that they have no competing interests.

## Authors’ contributions

VK premeditated and carried out the extraction of the *Paederia foetida* Linn leaves. VK, MM, DA, AV, AA, ZAD, PWR and PCB carried out the biochemical estimations. VK, VM and FA analyses the statistical data and interpretation of histological analysis. All the authors are involved in the critical evaluation of the manuscript. All authors read and approved the final manuscript.

## Pre-publication history

The pre-publication history for this paper can be accessed here:

http://www.biomedcentral.com/1472-6882/14/76/prepub
